# Differences in Overweight and Obesity among Children from Migrant and Native Origin: The Role of Physical Activity, Dietary Intake, and Sleep Duration

**DOI:** 10.1371/journal.pone.0123672

**Published:** 2015-06-01

**Authors:** Wim Labree, Dike van de Mheen, Frans Rutten, Gerda Rodenburg, Gerrit Koopmans, Marleen Foets

**Affiliations:** 1 Institute of Health Policy and Management, Erasmus University, Rotterdam, The Netherlands; 2 IVO Addiction Research Institute, Rotterdam, The Netherlands; 3 Erasmus MC, University Medical Center, Rotterdam, The Netherlands; 4 Department of Health Promotion, Maastricht University, Maastricht, The Netherlands; National Institute of Agronomic Research, FRANCE

## Abstract

A cross-sectional survey was performed to examine to what degree differences in overweight and obesity between native Dutch and migrant primary school children could be explained by differences in physical activity, dietary intake, and sleep duration among these children. Subjects (*n*=1943) were primary school children around the age of 8–9 years old and their primary caregivers: native Dutch children (*n*=1546), Turkish children (*n*=93), Moroccan children (*n*=66), other non-western children (*n*=105), and other western children (*n*=133). Multivariate regressions and logistic regressions were used to examine the relationship between migrant status, child’s behavior, and BMI or prevalence of overweight, including obesity (logistic). Main explanatory variables were physical activity, dietary intake, and sleep duration. We controlled for age, sex, parental educational level, and parental BMI. Although sleep duration, dietary intake of fruit, and dietary intake of energy-dense snacks were associated with BMI, ethnic differences in sleep duration and dietary intake did not have a large impact on ethnic differences in overweight and obesity among children from migrant and native origin. It is suggested that future preventive strategies to reduce overweight and obesity, in general, consider the role of sleep duration. Also, cross-cultural variation in preparation of food among specific migrant groups, focusing on fat, sugar, and salt, deserves more attention. In order to examine which other variables may clarify ethnic differences in overweight and obesity, future research is needed.

## Introduction

Overweight and obesity have become a major concern for public health [1]. Disease symptoms that once were only present in overweight adults, nowadays are becoming more common at young age [2]. Overweight in childhood often develops into obesity in adulthood. In addition, when overweight parents are nurturing children of their own, these children have a higher chance of developing overweight or obesity themselves, as parental Body Mass Index (BMI) is a predictor of their child’s BMI [3].

Due to the growing prevalence of childhood overweight and obesity, worldwide, and due to the fact that obesity is the fifth leading risk for global deaths, the World Health Organization (WHO) has recognized childhood obesity as one of the most serious challenges in public health of the 21^st^ century [4]. Besides the long-lasting adverse physical, psychological, and social health consequences, childhood obesity is also responsible for a substantial economic burden [5–6].

In general, overweight is the result of an excess of energy intake on energy expenditure, during a longer period of time [7–8]. However, whereas this definition looks quite simple, the etiology of overweight and obesity is complex and makes it challenging to develop effective preventive programmes and strategies [9]. Although the energy balance is determined by biologic, genetic, environmental, and behavioral factors, recent studies indicate that the overweight epidemic is more likely due to the latter [10–12]. Examples of these behaviors are physical exercise or sedentary behavior, food habits or dietary intake, and sleep duration.

According to a European review of the literature, children from migrant origin are more at risk of overweight and obesity than native children [13]. A recent study from The Netherlands showed that overweight and obesity are significantly more prevalent among migrant children from non-western descent than among native children and children from western descent [14]. Dutch prevalence rates of overweight and obesity are especially alarming among children in the two residing largest migrant groups: those from Turkish and Moroccan descent [15].

Effective prevention programmes and treatment strategies are necessary for these specific migrant groups. These particular interventions can only be adequately designed, if specific lifestyle behaviors that influence the elevated risk among these migrants are identified [16].

It is generally agreed that migration to developed countries seems to increase the risk of overweight and obesity [17]. The socio-economic status of migrants is lower than that of the native population, which may influence this risk [18]. Also, this increased risk can be caused by alterations in physical activity, for example, leading to a more sedentary way of life, and changes in dietary intake, resulting in westernized dietary patterns [19]. Additionally, recent attention has been paid to the independent influence of sleep on overweight and obesity [20–22]. Differences in sleep duration between primary school children from migrant and non-migrant origin have not been investigated earlier. However, a recent study among preschool children in Italy shows higher sleep durations in natives, as compared to migrants [23].

In The Netherlands, percentages in overweight and obesity among Turkish children (28%) and Moroccan children (26%) are about two times higher than among native children (13%). Although recent rates from The Netherlands show that overweight and obesity prevalences in children, overall, are declining, Turkish children show a stabilizing trend [24].

This study focuses on differences in overweight and obesity between native and migrant primary school children in The Netherlands. Migrant background is thought to explain ethnic differences in overweight and obesity among children through differences in behaviors, associated with overweight and obesity, which might be modifiable: physical activity, dietary intake (fruit, vegetables, sweet beverages, snacks), and sleep duration. The conceptual model of this study is presented in Fig 1.

**Fig 1:** Conceptual model. The influence of physical activity, dietary intake, and sleep duration on overweight and obesity.

## Materials and Methods

### Background study

A cross-sectional study was performed in the framework of the IVO Nutrition and Physical Activity Child CohorT (INPACT) study. The INPACT study is a collaborative project between the IVO Addiction Research Institute, and the Institute of Health Policy and Management, which is a department of the Erasmus University Rotterdam. In this project, the developmental trajectory of weight in Dutch primary school children was addressed, starting when they were 8–9 years old. The current study was based on the first data collection in the school year of 2008/2009.

### Study population

Data have been collected from parent-child dyads at primary schools, located in the cities and adjacent areas of Eindhoven and Rotterdam. Eindhoven is the fifth largest city in The Netherlands with about 200.000 residents and Rotterdam is the second largest Dutch city with about 600.000 residents. Children from different migrant backgrounds live and attend to school there.

Schools were invited for participation in this project by means of a letter in which research aim, background, and relevance were explained. Schools were excluded if they were participating in a current prevention program, aimed at overweight, as this might influence the measurements.

All parents received a letter, which provided information about this research project. In order to stimulate participation among the two largest migrant groups, Turkish and Moroccan parents received a letter in their native language. Also, they could receive assistance in this language by interpreters, while filling out the questionnaires, during specific consultation hours or by phone. Finally, of the 3162 invited parent-child dyads, 1943 dyads (61.5%) decided to participate in the study. Subjects at baseline were 8–9 years old school children. Participation in this study was on the basis of informed consent of the primary caregivers.

The study was approved by the medical ethics committee of the Erasmus MC, University Medical Center Rotterdam.

### Measurements

The primary caregiver of the child, mostly the mother, was asked to fill out the questionnaire. The questionnaire included questions on the child’s age and sex. Also, migrant background was asked. Children were considered as having a migrant background, when at least one of their parents was born outside The Netherlands, according to current practice in The Netherlands by Dutch Statistics [25]. Similar, based on this practice, five groups in our sample can be distinguished: native Dutch children (*n* = 1546), children with a Turkish background (*n* = 93), children with a Moroccan background (*n* = 66), and two supplementary groups, containing children from a range of countries, one with children from non-western origin (*n* = 105) and one with children from western origin (*n* = 133).

Apart from that, the questionnaire consisted of questions regarding both the weight and height of the parents, and regarding their socio-economic status, as defined by educational level. Questions were included on the education of both the mother, and the father. We determined the educational level by taking into account the parent that achieved the highest level, divided into three categories: low (primary school, lower vocational or general education), middle (secondary school, intermediate vocational school), and high (higher vocational school or university).

#### Outcome measures

Outcome measures are the mean BMIs of the children and the prevalence of overweight, including obesity, in each of the five groups. BMI, calculated as weight in kilograms divided by the square of height in meters, was used to assess weight status. Anthropometric measurements for the children were carried out by trained raters. Children were measured at school according to standard procedures in light clothing without shoes, to the nearest 0.1 kg and 0.1 cm. Weight was measured with an electronic flat scale (Seca 840; Beenhakker, Rotterdam, The Netherlands) and height was measured with a mobile measuring ruler (Seca 214; Beenhakker, Rotterdam, The Netherlands).

Apart from inclusion in our descriptive statistics, we excluded children with missing BMI scores and parent-child dyads of underweight children (*n* = 120), categorized on base of the International Obesity Task Force (IOTF) standard. The IOTF has developed an international reference standard to define weight categories in children [26]. This standard was used to divide the children into three categories: (1) underweight, (2) normal weight and (3) overweight, including obesity.

#### Child’s physical activity

To assess the children’s physical activity level, a questionnaire was used, based on a recognized method by the National Institute for Public Health and the Environment and by the local Public Health Services [27]. This questionnaire followed Welk and colleagues [28], who suggested to ask for various types of physical activity in specific key places, in terms of duration, and in terms of frequencies.

The primary caregiver had to write down how often, based on a normal week, children (1) went to school by foot or by bicycle (active transport), (2) played inside or outside, and (3) participated in a sport or at a sport club.

Based on the answers, as expressed in durations and frequencies, we calculated the average amount of minutes that the child spends on physical activity per day.

#### Child’s dietary intake

To ascertain the children’s dietary intake with regard to specific food categories, we made use of Food Frequency Questionnaires [29–30]. Four food categories were included: fruit (fresh, bottled, canned), vegetables (raw, cooked), sugar-sweetened beverages, and energy-dense snacks, such as potato crisps, candies, or chocolates.

The primary caregiver had to write down, based on an average week, how many days their children consumed products in these food categories. The answering scale included 8 categories, ranging from “none or less than 1 day a week” to “7 days a week”. Also, these caregivers had to score on such a day the number of fruit pieces, vegetable spoons (one spoon equals 50 grams), sweet beverage glasses, and snack pieces.

Total food consumption of the child with regard to these four food categories has been calculated and expressed in portions per day (pieces, grams, glasses, pieces).

#### Child’s sleep duration

The children’s sleep duration was measured by two items. The primary caregiver had to fill in the time that their children went to bed and awoke on an average school day. The answering scales of both questions consisted of time categories with intervals of half an hour. Also, two more broader time categories were used with an option “earlier than” or “later than” a specific time (e.g., “earlier than 6 am” or “later than 10.30 pm”). An extra half an hour was added or subtracted, in case a primary caregiver made use of these categories. The average amount of minutes that the child sleeps per night during a normal school week has been calculated.

### Analysis

Bivariate correlations (Pearson and Spearman correlation coefficients) were calculated to determine the relationships between behaviors (child’s physical activity, dietary intake, and sleep duration) and the dependent variables (child’s BMI and prevalence of overweight, including obesity), as well as the relationships between behaviors.

Multivariate linear regression was used to examine whether the relation between migrant background and child’s BMI could be explained by physical activity, dietary intake, and sleep duration. In addition, logistic regression was used to investigate whether ethnic differences in the prevalence of overweight, including obesity, could be explained by differences in behavior. Because both age and sex of the child, and educational level and BMI of the parents might influence overweight and obesity, the analyses controlled for these variables.

Four models were tested. In the first model, we tested the association between migrant status and BMI, adjusting for age, sex, parental educational level, and parental BMI. In the following three models, we included sleep duration, dietary intake, and physical activity. The order of adding these variables depended on the bivariate correlations, starting with the child’s behavior, which correlated most with BMI and the prevalence of overweight, including obesity, and ending with the behavior, which correlated least with these dependent variables. Missing values were omitted. Data were analysed by means of SPSS (version 19.0).

## Results

Table 1 displays the characteristics of our research sample per group (*n* = 1943). The upper part of this table shows mean age, percentages of boys and girls, educational level of the parents, and maternal and paternal BMI, in each group. The educational level of the parents of Turkish, Moroccan, and of the other non-western children was lower than that of the native Dutch children and the non-native western children. Additionally, BMIs of the mothers and fathers of Turkish and Moroccan children were significantly higher than those of the other parents (*p*<.05).

**Table 1:** Sample characteristics.

	Dutch (*n* = 1546)	Turkish (*n* = 93)	Moroccan (*n* = 66)	non-western (*n* = 105)	western (*n* = 133)
Age, M (SD) [missing]	8.2 (0.45) [4]	8.6 (0.67) [1]	8.5 (0.61) [1]	8.4 (0.63) [3]	8.3 (0.52) [2]
Boys, *n* (%)	778 (50.3)	38 (40.9)	36 (54.5)	44 (41.9)	74 (55.6)
Girls, *n* (%)	768 (49.7)	55 (59.1)	30 (45.5)	61 (58.1)	59 (44.4)
Educational level parents, %					
- Low	12.5	42.4*	34.5*	26.4*	13.9*
- Medium	39.7	37.6*	37.9*	35.2*	32.8*
- High [missing]	47.9 [23]	20.0* [8]	27.6* [8]	38.5* [14]	53.3* [11]
Mother’s BMI (kg/m^2^), [missing]	24.2 (3.9) [194]	25.5 (4.4)* [15]	25.7 (4.0)* [16]	24.5 (4.0) [39]	23.5 (3.1) [33]
Father’s BMI (kg/m^2^), [missing]	25.7 (3.1) [194]	27.3 (3.3)* [15]	26.8 (2.9)* [16]	25.2 (3.2) [39]	26.1 (3.2) [33]
Child’s physical activity level per day, minutes M (SD) [missing]	67.9 (21.0) [8]	38.0 (18.7)* [2]	56.9 (26.8)* [4]	41.1 (18.7)* [3]	62.0 (21.4)* [3]
Child’s fruit intake per day, pieces M (SD) [missing]	1.1 (0.6) [6]	1.3 (1.0)* [1]	1.4 (0.9)* [3]	1.2 (0.7)* [2]	1.3 (0.7)* [2]
Child’s vegetables intake per day, grams M (SD) [missing]	67.6 (34.8) [12]	75.9 (71.7)* [1]	84.9 (57.3)* [1]	72.7 (47.2)* [1]	72.4 (42.8)* [3]
Child’s sweet beverage intake per day, glasses M (SD) [missing]	1.4 (0.8) [3]	1.0 (0.6)* [2]	1.5 (1.1)* [1]	1.2 (0.9)* [1]	1.3 (0.8)* [3]
Child’s snack intake per day, pieces M (SD) [missing]	2.1 (1.1) [17]	1.6 (1.2)* [2]	1.5 (0.9)* [2]	1.6 (1.2)* [4]	1.9 (1.4)* [2]
Child’s sleep duration per night, minutes M (SD) [missing]	670.1 (27.7) [42]	645.5 (35.4)* [4]	645.3 (34.9)* [4]	654.8 (33.2)* [6]	657.5 (32.5)* [12]
Child’s BMI (kg/m^2^), M (SD)	16.4 (2.1)	19.0 (3.5)*	17.5 (2.6)*	17.6 (2.9)*	17.0 (2.7)*
overweight, including obesity, %	13.3	40.2*	24.2*	31.1*	22.0*
underweight, %	6.5	4.4*	1.6*	7.1*	8.2*

* *p*<0.05

In the lower part of Table 1, the mean BMIs of the children, the percentages of both overweight, including obesity, and of underweight, the child’s physical activity, dietary intake with regard to our four food categories, and sleep duration are presented. Overall, mean BMI scores differed between the groups of children (*p*<.05). Dutch children had the lowest BMI score (mean = 16.4 kg/m^2^; SD = 2.1). All children from migrant descent had higher BMI, especially Turkish children (mean = 19.0 kg/m^2^; SD = 3.5). Also, among migrant groups the prevalence of overweight, including obesity, were highest. Turkish and Moroccan children show the lowest prevalence of underweight, as compared to the other groups of children.

Child’s physical activity level in native Dutch children was higher than the physical activity level in migrant children (*p*<.05). Overall, Turkish children showed the lowest levels of physical activity, followed by other non-western, Moroccan, and other western children.

Although differences in dietary intake between children were relatively small, child’s fruit and vegetables intake was significantly lowest in Dutch children. Children in all migrant groups displayed higher fruit and vegetables consumption. Moroccan children scored highest in fruit intake per day (mean = 1.4 pieces per day; SD = 0.9) and vegetables intake per day (mean = 84.9 grams per day; SD = 57.3). Also, the consumption of sugar-sweetened beverages and energy-dense snacks was lower in migrants than in natives, except in Moroccan children.

Child’s sleep duration between the groups of children differed significantly (*p*<.05). Dutch children had the highest sleep duration, more than 11 hours (mean = 670.1 minutes per night; SD = 27.7). Also, all migrant children slept less than 11 hours per night, especially Turkish and Moroccan children. Differences between groups of children varied from 24.8 minutes to 12.6 minutes sleep per night.

Table 2 presents bivariate correlations between the behaviors and the dependent variable, as well as correlations between the behaviors. Less sleep, low fruit intake, and more energy-dense snack consumption correlated with higher BMIs and higher prevalence of overweight and obesity. Only dietary intake between some food categories correlated. Positive relationships were found between fruit and vegetables, and between sweet beverages and energy-dense snacks. Negative relationships were found between fruit and sweet beverages, and between vegetables and energy-dense snacks.

**Table 2:** Bivariate correlations.

	Physical activity level	Dietary intake (fruit)	Dietary intake (vegetables)	Dietary intake (sweet beverages)	Dietary intake (energy-dense snacks)	Sleep duration
Physical activity level	1					
Dietary intake (fruit)	.042 (*p* = .088)	1				
Dietary intake (vegetables)	.035 (*p* = .156)	.268* (*p* = .000)	1			
Dietary intake (sweet beverages)	-.009 (*p* = .713)	-.083* (*p* = .000)	-0.38 (*p* = .094)	1		
Dietary intake (energy-dense snacks)	-.040 (*p* = .110)	-.007 (*p* = .765)	-.103* (*p* = .000)	.172* (*p* = .000)	1	
Sleep duration	.001 (*p* = .968)	.017 (*p* = .458)	.009 (*p* = .687)	-.005 (*p* = .835)	-.023 (*p* = .323)	1
BMI child	-.047 (*p* = .056)	-.049* (*p* = .033)	-.040 (*p* = .086)	.019 (*p* = .410)	.094* (*p* = .000)	-.158* (*p* = .000)
overweight, including obesity	-.042 (*p* = .054)	-.046* (*p* = .049)	-.006 (*p* = .786)	.038 (*p* = .103)	.072* (*p* = .002)	-.091* (*p* = .000)

* *p*<0.05; (*n* = 1823)

In the regression analyses, we tested four models in Table 3 and Table 4 with sleep duration added in model 2 (highest coefficient), dietary intake added in model 3 (intermediate coefficient), and physical activity (lowest coefficient) added in model 4.

**Table 3:** Predictors of BMI child: results of multivariate regression analyses.

Variables	Model 1		Model 2		Model 3		Model 4	
	β	t	β	t	β	t	β	t
Age	0.08*	3.12	0.07*	2.75	0.08*	2.81	0.07*	2.77
Sex girl	0.06*	2.20	0.06*	2.45	0.07*	2.53	0.07*	2.65
Background								
- Turkish	0.24*	9.01	0.24*	9.05	0.23*	8.60	0.23*	8.65
- Moroccan	0.09*	3.14	0.08*	2.96	0.07*	2.44	0.07*	2.50
- non-western	0.05*	2.03	0.04	1.53	0.03	1.21	0.03	1.23
- western	0.00	0.01	0.01	0.45	0.01	0.51	0.01	0.52
Educational level								
- middle	-0.03	-0.72	-0.02	-0.43	-0.02	-0.46	-0.02	-0.48
- high	-0.00	-0.10	-0.01	-0.12	-0.01	-0.29	-0.02	-0.33
BMI mother	0.17*	6.11	0.16*	6.09	0.17*	6.16	0.17*	6.21
BMI father	0.18*	6.78	0.18*	6.74	0.18*	6.67	0.18*	6.66
Sleep duration			-0.12*	-4.46	-0.12*	-4.66	-0.12*	-4.71
Dietary intake (fruit)					-0.04	-1.28	-0.03	-1.23
Dietary intake (vegetables)					-0.04	-1.47	-0.04	-1.50
Dietary intake (sweet beverages)					0.01	0.40	0.01	0.38
Dietary intake (snacks)					0.05*	1.96	0.06*	2.04
Physical activity level							-0.03	-1.20
adjusted R^2^	0.17		0.19		0.20		0.20	
R^2^ change	0.17*		0.02*		0.01*		0.00	

* *p*<0.05

**Table 4:** Predictors of overweight and obesity: results of logistic regression analyses.

Variables	Model 1		Model 2		Model 3		Model 4	
	B	OR (95% CI)	B	OR (95% CI)	B	OR (95% CI)	B	OR (95% CI)
Intercept	-8.47*	0.00*	-4.66*	0.01*	-4.08*	0.02*	-4.09*	0.02*
Age	0.57*	1.59* (0.72–1.55)	0.37*	1.38* (0.70–1.51)	0.35*	1.36* (0.70–1.53)	0.34*	1.34* (0.70–1.53)
Sex girl	0.61*	1.83* (1.26–2.66)	0.62*	1.86* (1.28–2.71)	0.62*	1.86* (1.28–2.70)	0.63*	1.87* (1.28–2.74)
Background								
- Turkish	1.62*	5.07* (2.48–10.36)	1.61*	4.99* (2.42–10.30)	1.40*	4.05* (1.92–8.54)	1.41*	4.09* (1.94–8.66)
- Moroccan	0.89*	2.42* (0.99–5.87)	0.87*	2.32* (0.93–5.60)	0.86*	2.29* (0.76–4.94)	0.84*	2.23* (0.77–4.98)
- non-western	0.94*	2.56* (1.01–6.54)	0.82	2.18 (0.88–5.92)	0.66	1.93 (0.73–5.08)	0.66	1.94 (0.73–5.13)
- western	0.23	1.26 (0.51–3.10)	0.13	1.14 (0.46–2.84)	0.05	1.05 (0.42–2.66)	0.06	1.06 (0.42–2.68)
Educational level								
- middle	-0.29	0.75 (0.43–1.31)	-0.24	0.79 (0.45–1.38)	-0.22	0.80 (0.45–1.41)	-0.23	0.80 (0.45–1.41)
- high	-0.22	0.80 (0.46–1.38)	-0.19	0.83 (0.48–1.43)	-0.28	0.76 (0.43–1.33)	-0.28	0.76 (0.43–1.32)
BMI mother	0.08*	1.08* (1.03–1.13)	0.08*	1.08* (1.03–1.13)	0.08*	1.08* (1.03–1.13)	0.08*	1.08* (1.03–1.13)
BMI father	0.15*	1.16* (1.09–1.23)	0.15*	1.16* (1.09–1.23)	0.14*	1.15* (1.09–1.22)	0.14*	1.15* (1.09–1.22)
Sleep duration			-0.01*	0.99* (0.98–1.01)	-0.01*	0.99* (0.98–1.00)	-0.01*	0.99* (0.98–1.00)
Dietary intake (fruit)					-0.02	0.98 (0.97–1.06)	-0.02	0.98 (0.97–1.06)
Dietary intake (vegetables)					-0.00	1.00 (0.99–1.01)	-0.00	1.00 (0.99–1.01)
Dietary intake (sweet beverages)					0.02	1.02 (0.96–1.06)	0.02	1.02 (0.96–1.06)
Dietary intake (snacks)					0.02	1.02 (0.95–1.04)	0.02	1.03 (0.95–1.14)
Physical activity level							-0.00	0.99 (0.99–1.00)
Nagelkerke R^2^	0.14		0.16		0.16		0.16	
R^2^ change	0.14*		0.02*		0.00		0.00	

* *p*<0.05

The first model tested the influence of migrant status, controlled for age, sex, parental educational level, and parental BMI. Taking into account these variables, Turkish, Moroccan, and non-western children, showed higher BMIs and prevalences of overweight and obesity, as compared to Dutch natives. This was not the case for western children.

Adding sleep duration (model 2) has led to a significant R^2^ change in both regressions. Ethnic differences between migrant children, compared with their indigenous counterparts, as expressed in a constant or slightly diminishing β (multivariate regression) and B (logistic regression) between model 1 and 2, were hardly explained. The unstandardized coefficient (B) of sleep duration in the multivariate regression was -0.008 (not in table), implying that, for example, an extra half an hour of sleep, which is about the highest observed mean difference across groups of children, will lead to a BMI decrease of 0.24 (30 minutes*-0.008). Similarly, the OR shows that more sleep slightly decreases the probability of overweight, including obesity.

Dietary intake of snacks (model 3) has led to a significant R^2^ change in the multivariate regression and not in the logistic regression, whereas β and B of migrant children, as compared to native children, did not change substantially. The unstandardized coefficient (B) of snack intake in the multivariate regression was 0.014 (not in table), implying that one more snack each day will lead to a BMI increase of 0.01. The impact of sleep duration (B and OR) did not change.

After including physical activity level (model 4) in the regression analysis, there was no significant R^2^ change and β and B did not change substantially. The impact of sleep duration (B and OR) and snack intake (B) did not change.

## Discussion

Objective of this study was to explain differences in overweight and obesity among children from migrant and native origin. We found that low sleep duration, low fruit intake, and high snack intake were associated with higher BMIs and higher prevalence of overweight and obesity. Both sleep duration, and snack intake explained BMI to some extent. However, ethnic differences in sleep duration and dietary intake only slightly contributed to explaining the observed ethnic differences in BMI or in the prevalence of overweight and obesity between native Dutch and migrant children.

Children from migrant descent showed the lowest sleep duration. Also, migrant children displayed significantly lower levels of physical activity. In this study, sleep duration was associated with BMI and with overweight and obesity prevalence. In contrary to our expectations, physical activity was not associated with BMI and with the prevalence of overweight and obesity. The results with respect to sleep duration are in line with recent European research, which indicates that sleep duration is associated with BMI in children, independent of physical activity of the children, and demographic variables, such as socio-economic position [31]. Still, ethnic differences in sleep did hardly explain overweight and obesity differences.

Our counterintuitive findings concerning the role of physical activity can be put into perspective by a recent systematic review, in which the relationship between physical activity level and overweight and obesity is discussed. Results point out that, apart from other health benefits, higher physical activity levels do not always result in lower BMIs, at least among adolescents [32]. Perhaps, therefore, it is not surprising we were unable to explain ethnic overweight and obesity differences. More research is needed at this point.

Concerning dietary intake, differences between groups of children were significant. All migrant groups displayed higher fruit and vegetables intake and lower energy-dense snack consumption. In this study, high fruit intake and low energy-dense snack intake did lead to lower BMIs. However, ethnic variations in overweight and obesity were hardly explained by ethnic variations in dietary intake.

Similar to physical activity, the relationship between fruit intake and the development of overweight and obesity is subject to discussion. The Mediterranean diet pattern, consisting of more vegetables, more fish, and more olive oil, is often regarded as healthy. However, dietary habits of some ethnic groups in Europe are likely to become less healthy as individuals increase consumption of processed foods that are energy dense and contain high levels of fat, sugar, and salt. Therefore, particular preparation methods among specific migrant groups, focusing on fat, sugar, and salt, deserve more attention, as such products often are added to the healthy dietary components of the native diet [33]. These mixed food habits are emerging mainly amongst younger people, probably as the consequence of acculturation processes, which increases the risk of overweight and obesity [34]. Therefore, overweight and obesity research in relation to dietary intake should also include energy density, energy content, and preparation methods of food.

Further, the use of specific terms in our questionnaires may have influenced our results. For example, the different units of measure (pieces, grams, glasses, pieces) may have caused some confusion, both among natives, and among migrants. At the same time, it is difficult to determine a standard unit of measure for various food categories. In addition, the use of the words sugar-sweetened and energy-dense may evoke social desirability bias.

As said before, the etiology of overweight and obesity is complex. This study only focused on behaviors associated with overweight and obesity, leaving out genetic and biological aspects. Apart from the role of our studied behaviors, physical activity, dietary intake, and sleep duration, we did not include sedentary behavior, such as watching television or playing computer games. Research should also include this more passive behavior.

Concerning the measurements of the behaviors in this study, the cross-cultural validity of our instruments may be questioned. Migrants and non-migrants may differ in their answering patterns, leading to cultural bias. In the literature, no evidence on the validity of these questionnaires among migrants was found. Therefore, we strongly recommend that future research should pay attention to this specific issue.

Strength of this study is the measurement of child weight and height by trained raters, rather than by parental report. We could also control for parental BMI. Unfortunately, parental weights and heights were assessed by self-reports, which may lead to socially desirable answers. Our results may have been biased by these self-reports.

In this study, we assessed physical activity, dietary intake, and sleep duration of the children by means of parental reports. Apart from the latter, validated instruments to measure these behaviors were used. We did not use self-reports by the children because they experience more problems with memory tasks regarding physical activity at this age, as compared to adults [35]. However, estimates of child’s intake of food by parents might not always agree with the actual dietary intake, as parents may not know what their children eat outside the home environment. Perhaps, it would have been better to ask children themselves to fill out this questionnaire, as some authors suggest that children aged 8–11 years are more accurate reporters of Food Frequency Questionnaires than their parents [36].

Further, our questionnaire only measured sleep duration by two questions: the time children went to bed and the time children awoke. Primary caregivers had to fill out the questions. We did not use self-reports by the children. Although these caregivers often know what time the child goes to bed, they may not know if the child actually is asleep. A more objective method might have been the use of physiological measurements [37].

As sleep duration is related to BMI and overweight and obesity prevalence, we suggest that future overweight and obesity strategies include the role of sleep duration in their prevention activities. This is a potentially modifiable risk factor for overweight and obesity, which is relatively easy for parents to implement and to control in their home environments, in order to prevent overweight and obesity, not only among children from migrant origin, but among all children.
